The article "Electrochemical Intelligent Recognition of Mineral Materials Based on Superpixel Image Segmentation" was retracted in 2023. Reasons: signs of a paper mill; suspected computer-generated content; unreliable results or conclusions; concerns about the data.

# Electrochemical Intelligent Recognition of Mineral Materials Based on Superpixel Image Segmentation

**DOI:** 10.1155/2022/6755771

**Published:** 2022-06-15

**Authors:** Weiping Liu, Fangzhou Jin

**Affiliations:** Department of Fundamental Subjects, Wuchang Shouyi University, Wuhan 430064, China

## Abstract

In order to study the needs of identifying rock thin-section samples by manual observation in the field of geology, a method of electrochemical intelligent recognition of mineral materials based on superpixel image segmentation is proposed. The image histogram of this method can be used to represent the distribution of each pixel value of the image. This interval is consistent with the number of pixels in the method. And using the experiment, the CPU used in the experiment is Intel® Core™ i7-8700 3.2 GHz, the memory is 16 GB, and the GPU is NVIDIA GeForce GT × 1080 Ti, which ensures the accuracy of the experiment. Based on all the experimental results, it can be seen that after the two-stage processing of the designed superpixel algorithm and the region merging algorithm, the final sandstone slice image segmentation results are close to the results of manual labeling, which is helpful for the subsequent research on sandstone component identification. The feasibility of this method was verified.

## 1. Introduction

Sandstone is one of the most widely distributed reservoir rocks in the world. The identification of sandstone thin sections is of great significance in the process of oil and gas resource exploration. At present, the traditional identification methods are time-consuming and labor-consuming, and the identification standards are not unified. Therefore, the processing and analysis of sandstone thin-section images by computer has practical application value [1]. According to the investigation and analysis, the algorithm processing flow of segmenting the image before recognition is designed. Aiming at the existing problems, two key technologies of sandstone slice image segmentation and component recognition are studied [2]. The pixel blocks obtained by Xianyi et al. through the above steps are superpixels. The method is performed on the BSDS500 dataset, and the experimental results show that the boundary recall (BR) and achievement segmentation accuracy (ASA) are 95.0% and 96.3%, respectively. Furthermore, the proposed method has better performance in terms of efficiency (30 fps). Comparative experiments show that superpixel boundaries not only have good adhesion to the original textures and contours of salient objects, but also can effectively reduce redundant superpixels in uniform regions [3].

VGGNet is a commonly used network model at present. The model won the runner up of ImageNet competition in 2014, which proves that increasing the depth of the network can improve the performance of the model to a certain extent. VGGNet all uses 3 × 3 convolution kernel and 2 × 2. The maximum pooling strategy is to divide the network structure into multiple segments, in which multiple convolution layers are connected in series, and a pooling layer is added between the two segments for downsampling. VGGNet has a deeper network structure than AlexNet. At present, 16-layer or 19-layer VGGNet is widely used. So, the subsequent classical models only use 3 × 3 or 1 × 1 convolution kernel to extract features. VGGNet also adopts the pretraining strategy. First, train a simple model, and then use its parameters to train the complex model so as to speed up the convergence speed of the training model. VGGNet not only increases the number of network layers, but also increases the amount of model parameters, but most of the parameters come from the full connection layer, which also promotes the related research of many lightweight neural network structures [4]. Image histograms are widely used in various fields of image processing, especially threshold segmentation, color-based image retrieval, and image classification, due to their small computational cost and many advantages of image translation, rotation, and scaling invariance.

The article "Electrochemical Intelligent Recognition of Mineral Materials Based on Superpixel Image Segmentation" was retracted in 2023. Reasons: signs of a paper mill; suspected computer-generated content; unreliable results or conclusions; concerns about the data.

GoogLeNet surpassed VGGNet to win the championship in the 2014 ImageNet competition. The concept of inception structure is proposed in the model. Convolution of 1 × 1, 3 × 3, and 5 × 5 and maximum pooling of 3 × 3 are paralleled in the same structure. Which increases the network width and improves the ability of the model to extract multiscale features. The results of all convolution operations in the inception structure are processed with the ReLU function and then spliced into a characteristic graph as the output. The idea of modular design in GoogLeNet is convenient and flexible to adjust the network depth. In order to avoid the disappearance of gradient, the network also adds two auxiliary classifiers in the middle layer for back-propagation gradient. Finally, the network adopts the global average pooling strategy and connects a full connection layer to flexibly adjust the output dimension [5]. It has been proved that the image recognition accuracy of GoogLeNet is higher than that of AlexNet, and the network structure is deeper than that of AlexNet, but the amount of parameters is 1/12 of the latter.

In view of the complexity of particle segmentation in the microscopic image of sandstone thin section, the existing segmentation methods are difficult to achieve satisfactory segmentation results. In order to overcome the shortcomings of the existing segmentation methods, this paper takes the multiangle orthogonal polarization microscopic image as the input and uses the different interference colors of sandstone mineral particles under different-angle polarization to improve the contrast between adjacent particles so as to accurately locate the boundary of sandstone particles. In addition, convolutional neural network is designed and trained to extract the semantic features of mineral particle image and identify different sandstone mineral types so as to improve the accuracy of segmentation, as shown in Figure 1.

The article "Electrochemical Intelligent Recognition of Mineral Materials Based on Superpixel Image Segmentation" was retracted in 2023. Reasons: signs of a paper mill; suspected computer-generated content; unreliable results or conclusions; concerns about the data.

## 2. Literature Review

Zhang et al. said that in the field of computer vision, image segmentation refers to dividing a digital image into multiple image subregions [6]. Jia believes that the methods used in the current research on sandstone slice image segmentation can be roughly divided into three categories: edge-based method, which recognizes the crystal boundary through the sharp change of pixel brightness or intensity at the edge. Based on the region method, the pixels are divided into multiple subregions by region growth method and clustering method. The energy-based method usually defines the energy function and then minimizes the energy function to extract the particles in stages [7].

Region-based methods usually cluster adjacent pixels with similar attributes into regions to identify particles. The edges produced by this method may be inaccurate. The research method is based on superpixel algorithm, which is a region-based segmentation method. The following focuses on the relevant research status of region based method. Alipour et al. proposed a color clustering slice mineral segmentation method based on incremental learning, which extracts 12-dimensional feature vectors for each pixel from RGB and its color space, automatically adjusts the number of cluster centers using the improved art algorithm, and clusters each pixel to the cluster center [8]. Huang et al. collected 155 slice images of 28 minerals for experiments and achieved 85.24% segmentation accuracy. However, the collected images contain less mineral particles and did not verify whether the algorithm is feasible for images containing a large number of particles [9]. In addition to the automatic image segmentation algorithm, it will help to improve the segmentation effect by adding the prior knowledge input manually and designing an interactive image segmentation method. Wei et al. proposed a semiautomatic image segmentation method based on seed region growth and used it for quantitative analysis of micro grain structure [10]. In their study, they used orthogonal polarized images of weathered sandstone samples at different angles as input and combined five images to enhance the hue difference between adjacent particles and pores. Kishorjit et al. believe that some seed points are manually set in the middle of the target particle area of the comprehensive image, and regional segments are created near each seed point; then the distance of feature space between adjacent areas is calculated, and the area near each seed point is iteratively classified into seed subareas of the same category so as to finally make the seed point area grow into subareas with uniform spectrum so as to complete the segmentation of weathered sandstone slice image [11]. Quan et al. developed interactive image segmentation software. Users can draw rough marks on the rock surface image to indicate the position of different mineral units in the image, and then the algorithm will segment the region based on the color uniformity of the region and detect the local target boundary so as to assist users in analyzing the rock image [12].

The article "Electrochemical Intelligent Recognition of Mineral Materials Based on Superpixel Image Segmentation" was retracted in 2023. Reasons: signs of a paper mill; suspected computer-generated content; unreliable results or conclusions; concerns about the data.

Superpixel segmentation is an image region oversegmentation algorithm, which divides the image into multiple irregular subregions according to the feature similarity between pixels. At present, SLIC, seeds, LSC, and other algorithms have better results. Taking the LSC (Linear Spectral Clustering) algorithm proposed by Egorova and Sergeyev as an example, the kernel function is designed to calculate the similarity measure based on the color similarity and spatial position proximity between pixels, and the superpixel segmentation results are obtained by iterative clustering [13]. NVIDIA researchers Varun et al. combined the superpixel algorithm with deep learning and proposed the SSN (Superpixel Sampling Networks) model so that the deep network can be trained end to end and produce superpixels, and its performance is better than the existing superpixel algorithms. Superpixel algorithm can be used to segment sandstone slice image. Shang et al. designed and developed a software system for sandstone microscopic image analysis [14]. Wang et al. believe that the system first uses SLIC superpixel algorithm to divide the image into hundreds of superpixels with regular shape and then measures the similarity between adjacent super pixels and combines the oversegmented regions so that the final generated superpixels contain complete mineral particle regions [15]. In the follow-up work of their team, they proposed a SLIC algorithm based on multiangle images; that is, using the sandstone image taken under the multiangle polarizing microscope, first generate the superpixels with boundary adhesion and oversegmentation, then extract the boundary, color, and texture features of each super pixel, and then merge the super pixels twice, and finally segment the more obvious feldspar, quartz, and other particles in the sandstone.

The article "Electrochemical Intelligent Recognition of Mineral Materials Based on Superpixel Image Segmentation" was retracted in 2023. Reasons: signs of a paper mill; suspected computer-generated content; unreliable results or conclusions; concerns about the data.

Identifying the classification of composition and structure in sandstone slice image is a necessary step to determine the genesis and properties of sandstone. At present, there is little research on sandstone slice image recognition. The usual method is to extract features from the image and then train the classifier to recognize the texture, category, source, and other properties of rocks.

## 3. Method

### 3.1. Introduction to Image Histogram and Histogram Equalization

The histogram of the image can be used to represent the distribution of each pixel value of the image [16]. Each cell has the number of pixels falling in this interval that is consistent with the range of the interval. The image histogram can graphically and intuitively display the occurrence frequency of each pixel in the image on different intensity values. If it is a gray image, the intensity range is [0 ∼ 255]. If it is a colored image, the image is generally separated into three RGB color channels, and each channel will have an image histogram. If there are two high points in the gray image histogram, that is, two gray levels of high ratio, there should be a binarization threshold between the two peaks. Histogram is the visual representation of image distribution. The abscissa of the histogram represents the type of image pixel value, which can be pixel gray value or RGB channel value [17]. The ordinate represents the number of features at the point, which can also be regarded as the proportion of the point feature in the whole image.

Histogram is a statistical relationship that represents the frequency of each gray level in a digital image. Histogram can give a general description of the gray range, that is, the frequency and distribution of each gray, as well as the average brightness and contrast of the whole image. The gray level histogram corresponds to a function about gray level. The abscissa of the histogram is a feature of the image, the gray level image is the gray level value, and the colored image is a channel value of the RGB channel. The ordinate represents the number of features at this point pr (*R*), which can also be regarded as the proportion of the point feature in the whole image. The distribution law of image features can be seen from the whole coordinate. Take the gray-scale image as an example. If the low gray-scale pixels are absolutely dominant in the histogram, the whole image will show a gray state. If the high gray-scale pixels account for the vast majority, the whole image will show a bright state [18].

The article "Electrochemical Intelligent Recognition of Mineral Materials Based on Superpixel Image Segmentation" was retracted in 2023. Reasons: signs of a paper mill; suspected computer-generated content; unreliable results or conclusions; concerns about the data.

The image is composed of pixels, so the histogram reflecting the pixel distribution can be used as an important tool of image processing. In practical applications, image histogram has effective and wide applications in image segmentation, feature extraction, and image matching. Histogram is also an important basis for adjusting image contrast. In the digital age, histogram can be said to be everywhere [19]. We can use the slender peak of the image histogram to judge which gray level the main information of the image is concentrated on, use the area between the two peaks of the image histogram to judge which gray level the background color is on, or use the peak valley to judge the gray level of the noise. Similarly, we can use the gray level expectation in the image to give an ideal binary boundary value. Even in hand painting, the main tone, background color, and the color range corresponding to the highlighted points are determined, which greatly reduces the difficulty of color matching.

Considering the continuous gray value, *R* represents the gray value of the original image, and its value range is [0, *L* − 1], where 0 represents black and white and *L* − 1 represents white. The new gray value obtained by the mapping function is represented by *s*, and each *s* corresponds to an *R*. *R* and *s* represent the gray value of the same pixel before and after mapping by the transformation function [20]. The transformation function is shown as follows:

(1) $$\begin{array}{c} s=T\left(r\right),\;0\leq r\leq L-1. \end{array}$$

Continuous random variable: in order to obtain the gray-scale mapping function of the algorithm, the gray-scale values of all pixels of an image are regarded as a group of random variables, and the range of variables is 0 to *L* − 1. The relationship between the values of random variables is described by their probability density function (PDF) [21]. Let *P*_*r*_ (*r*) and *P*_*s*_ (*s*) represent the PDF of random variables *R* and *s*, respectively. If *P*_*r*_ (*r*) and *t* (*t*) are known, the PDF of *s* after mapping function transformation is shown as follows:

(2) $$\begin{array}{c} P_{s}\left(s\right)=P_{r}\left(r\right)\left|\frac{dr}{ds}\right|. \end{array}$$

Since the histogram to be equalized is evenly distributed, its PDF is known, as shown in the following formula:

(3) $$\begin{array}{c} P_{s}\left(s\right)=\frac{1}{L-1}. \end{array}$$

Therefore, the following can be concluded that, as shown in the following formulae:

(4) $$\begin{array}{c} P_{r}\left(r\right)\left|\frac{dr}{dT\left(r\right)}\right|=\frac{1}{L-1}, \end{array}$$

(5) $$\begin{array}{c} \left|\frac{dT\left(r\right)}{dr}\right|=\left(L-1\right)P_{r}\left(r\right), \end{array}$$

(6) $$\begin{array}{c} T\left(r\right)=\left(L-1\right)\frac{d}{dr}\left[\int_{0}^{r}P_{r}\left(w\right)\text{d}w\right]. \end{array}$$

Finally, the transformation function of *T* (*T*) is obtained, which converts arbitrary PDF into uniform PDF, as shown in Figures 2 and 3.

The article "Electrochemical Intelligent Recognition of Mineral Materials Based on Superpixel Image Segmentation" was retracted in 2023. Reasons: signs of a paper mill; suspected computer-generated content; unreliable results or conclusions; concerns about the data.

It can be verified that the final conversion function *T* (*r*) satisfies both conditions (a) and (b). Discrete mapping function: the specific mapping applied to each pixel requires a discrete mapping function to map each pixel of the image. After the transformation function of continuous gray level, it can be applied to discrete situations. For discrete values, we deal with their discrete probability instead of PDF. In an image, the probability of occurrence of pixels with gray value of *n* can be roughly shown in the following formula:

(7) $$\begin{array}{c} P_{r}\left(r\right)=\frac{n_{k}}{MN}. \end{array}$$

The discrete form of transformation *T* (*r*) is shown as follows.

(8) $$\begin{array}{c} s_{k}=T\left(r_{k}\right). \end{array}$$

The advantages of histogram equalization algorithm are as follows: firstly, the gray value of new pixel points is obtained through the gray value mapping function, which can improve the clarity and contrast of the image and make the image details that users want more obvious. Especially when the pixel values of the image are concentrated in a certain cell, through this way of pixel value redistribution, the characteristic information of pixels can be more evenly and reasonably distributed in the whole image [22]. Thus, the pixel features of the image can be extended to enhance the image contrast. Histogram equalization algorithm is particularly suitable when dealing with images with several gray values of background and foreground in a certain area. Particularly for X-ray images, histogram equalization algorithm can improve the contrast and detail information of X-ray images, making the images easier for medical analysis.

### 3.2. MMTD Introduction

The intermediate logic calculus system is deduced according to the ternary semantics. The first value is marked as *t*, indicating positive, and the second value is marked as *f*, indicating negative [23]. The third value is represented by *m*, and the third value is the mediation state. Thus, {*T*, *m*, *f*} is the truth set of the mediation logic system. The fuzzy negative words reflecting fuzziness in the intermediate logic calculus system are expressed by “∼”. The truth degree word describing the difference between two life words is expressed by “<”. However, the original method of intermediary logic system does not have a quantitative research system for fuzzy phenomenon. For example, given predicate *Q*, *Q* (*Y*) can only qualitatively indicate that variable *y* has property *Q*, but the degree to which *y* has *Q* cannot be obtained. For another example, although the truth degree of *C* and *D* can be known from *C* < *D*, the difference between the truth degrees of *C* and *D* cannot be known according to the original intermediary logic system. Therefore, in terms of practicability, it is very necessary to study and establish the quantitative research method of intermediate truth system. MMTD is a numerical quantitative method. MMTD is a numerical quantitative method. In MMTD formula, the distance is expressed as follows.

(9) $$\begin{array}{c} d\left(a,b\right)={\left[\sum_{i=1}^{n}{\left(a_{i}-b_{i}\right)}^{2}\right]}^{1/2}. \end{array}$$

In the case of one dimension, it is shown as follows.

(10) $$\begin{array}{c} d\left(a,b\right)=\left|a-b\right|. \end{array}$$

MMTD is a method different from fuzzy mathematics and quantitative processing of fuzzy phenomena. Since Professor Hong Long founded the MMTD method in 2006, MMTD has been effectively applied in many fields and achieved successful results. Compared with pure fuzziness, MMTD has a solid theoretical and logical foundation [24]. Yang Xiaobin proposed a face recognition method based on MMTD; Zhou Ningning and others designed and implemented an image denoising and filtering algorithm based on MMTD; Zhou Ningning and Hong Long designed and implemented an evaluation method based on intermediate truth degree measurement; Wang Cen and others designed and implemented the search processing of knowledge reasoning based on MMTD: Yang Xiaolin proposed an image mosaic method based on MMTD. The successful applications in these different fields verify the effectiveness and feasibility of MMTD in dealing with fuzzy phenomena.

The article "Electrochemical Intelligent Recognition of Mineral Materials Based on Superpixel Image Segmentation" was retracted in 2023. Reasons: signs of a paper mill; suspected computer-generated content; unreliable results or conclusions; concerns about the data.

The image enhancement algorithm can increase the contrast of the image, whether it is the overall contrast or the local contrast, and can make some useful features of the image more prominent. The image after image enhancement is more in line with the visual characteristics of human eyes and easier for machine recognition.

Due to the limitation of image capture equipment or the existence of nonideal environment, many times, these images may need some degree of enhancement to meet people's visual requirements. Due to the limitation of external environmental conditions in the transmission process, the quality of the image is distorted, resulting in the information can not be read and recognized normally. In order to improve the visual effect of the image, highlight the interesting part of the image, and remove the unnecessary information, the image needs to be preprocessed. The operation process of preprocessing is called image enhancement [25]. After the enhanced image, the desired features of the user in the image are more obvious, the intuitive visual effect of the image is improved, and the improved image will be more suitable for a given occasion and application. The image enhancement algorithm purposefully emphasizes the global or local image characteristics so as to make the unclear part of the original image clearer, improve the difference between the characteristics of different parts in different regions of the image, weaken the unnecessary features in the application, remove the unwanted features of the image, and expand the gray level of the image so as to enhance the visual effect of the image on the human eye to meet the specific demand analysis. Image enhancement is a process of dealing with undesirable distortion caused by weak contrast, unwanted noise, inappropriate intensity saturation, blur effect, and so on and determining the hidden information contained in the image. The main purpose of image enhancement is to provide effective image preprocessing for image processing so that the preprocessed image is more suitable for later image processing algorithms than the original image. The image preprocessing effect of image enhancement can directly determine the quality of subsequent image analysis. Therefore, how to improve the effect of image enhancement is very important. At present, image enhancement technology has been widely used in public health and safety, medicine, industrial research, aerospace, and other fields [26].

The depth of convolutional neural network is closely related to the ability of feature expression. In order to further increase the depth of network structure, He et al. proposed ResNet model. The model won the championship in the ImageNet competition in 2015. The top-5 recognition error rate on the ImageNet dataset is 3.57%, even lower than the human eye recognition error rate. Simply stacking convolution layers to increase the depth will lead to gradient disappearance or gradient explosion, and the performance of the network may deteriorate with the increase of depth. He et al. proposed an assumption that when a simple convolution layer stacking leads to too deep network, if the feature extracted by one layer is already in the optimal state, the later layer should not change it, so the later layer should learn the ability of identity mapping. The module structure is shown in Figure 4.

## 4. Results and Analysis

The main content is to evaluate and analyze the advantages and disadvantages of the proposed algorithm and compare it with several classical superpixel algorithms. All images used in the experiment are selected from BSDS500 and SISD data sets, and the codes of the comparative experiment are implemented in Python [27].

The article "Electrochemical Intelligent Recognition of Mineral Materials Based on Superpixel Image Segmentation" was retracted in 2023. Reasons: signs of a paper mill; suspected computer-generated content; unreliable results or conclusions; concerns about the data.

### 4.1. AS-SLIC Algorithm Verification

Here, 20 images are selected from SISD data set for experiments to verify whether the proposed AS-SLIC algorithm can adaptively produce different numbers of superpixels. In the experiment, the SLIC algorithm is used as a control. The SLIC algorithm sets the compactness factor *M* = 30 and the expected number of superpixels *k* = 25. The experimental results are shown in Figure 5.

The experimental results show that the setting of parameter *K* makes the number of superpixels generated by SLIC algorithm more balanced. When the number of real regions is greater than the parameter value, there will be an undersegmentation problem. The number of superpixels generated by AS-SLIC algorithm has a certain correlation with the number of real regions and is always more than the number of real regions. This is because the number of real regions in sandstone slice image is related to the color histogram, and AS-SLIC algorithm uses the color histogram to dynamically adjust the number of superpixels. To sum up, AS-SLIC algorithm adaptively generates superpixels through image color features, omits parameter settings, and alleviates the problem of under segmentation to a certain extent [28]. The disadvantage of AS-SLIC algorithm is that there will be misjudgment when looking for the peak, which may cause a certain degree of oversegmentation.

### 4.2. Comparison of Superpixel Segmentation Algorithms

The AS-SLIC algorithm is compared with SLIC, SDDES, LSC, and QS algorithms. The parameter configuration of the algorithm in the experiment is as follows: the initial number of superpixels of SLIC algorithm is set to 50, the compactness factor is set to 30, and the number of iterations of the algorithm is 10. The compactness factor of AS-SLIC algorithm is set to 25, and the number of iterations of the algorithm is 10: the core size of QS algorithm is 13, the maximum distance is 17, and the color space ratio is 0.5.

The experiment is evaluated based on 200 training set images in BSDS500 and 20 orthogonal polarizing images of sandstone slices in SISD. The evaluation index in the table is the average score obtained by the algorithm on all images. When processing BSDS500 data sets, SEEDS algorithm has the highest boundary recall rate, mainly because the superpixel shape generated by this algorithm is irregular and has a high degree of fit to the edge, but the boundary accuracy of segmentation results is low. In the experiment based on SISD data set, the proposed AS-SLIC algorithm has the lowest hue value, which shows that this algorithm is more conducive to solve the undersegmentation problem than other algorithms. Compared with SLIC algorithm, the boundary recall rate of AS-SLIC algorithm is 0.9% higher than that of SLIC algorithm, indicating that the superpixel boundary fit degree is better than SLIC algorithm. Compared with other algorithms, AS-SLIC algorithm has higher *F*-measure value, which is mainly due to the improvement of boundary recall rate, which shows that this algorithm is more conducive to detecting object edges in the image. It is worth noting that the *F*-measure of AS-SLIC in BSDS500 is slightly lower than that of SLIC. The main reason is that the number of target areas in BSDS500 is generally small, and the number of superpixels generated by SLIC algorithm is relatively balanced. When the number of superpixels is less than the number of real areas in the image, there are fewer segmentation boundaries beyond the real boundary, so the precision value of SLIC algorithm is high. AS-SLIC is more prone to oversegmentation than SLIC algorithm, resulting in lower precision value than SLIC algorithm, so *F*-measure is lower than SLIC algorithm.

The article "Electrochemical Intelligent Recognition of Mineral Materials Based on Superpixel Image Segmentation" was retracted in 2023. Reasons: signs of a paper mill; suspected computer-generated content; unreliable results or conclusions; concerns about the data.

In terms of algorithm time complexity, AS-SLIC algorithm needs to traverse *N* pixels in each iteration in the clustering process, so the time complexity of clustering is *O* (*N*). At the same time, each iteration needs to count the color histogram of superpixels, and the time complexity of statistical histogram and peak searching is *O* (*N*). Therefore, the comprehensive time complexity of AS-SLIC algorithm is *O* (*N*), which is linearly related to the total number of image pixels. The processing resolution is 1392 × 1040.  The time complexity of QS algorithm is *O*, so it takes much more time than other algorithms. Among them, SEEDS algorithm runs the fastest. The proposed AS-SLIC algorithm is about twice as fast as SLIC algorithm, which is similar to LSC algorithm. The average time of the algorithm is shown in Table 1.

Experimental results show that the proposed AS-SLIC algorithm can adaptively produce superpixels that fit the local particle region and alleviate the undersegmentation problem of the traditional algorithm to a certain extent. Multi-image superpixel segmentation experiments based on sandstone slice single polarization and orthogonal polarization images show that the combination of sandstone slice images under the two light sources is helpful to produce more accurate segmentation results. Finally, the proposed superpixel merging algorithm can merge most of the superpixels belonging to the same debris particles into a complete region and solve the problem of superpixel oversegmentation to a certain extent. According to all the experimental results, after the two-stage processing of the designed superpixel algorithm and region merging algorithm, the final segmentation result of sandstone slice image is close to the result of manual annotation, which is helpful to the subsequent research of sandstone component recognition.

The article "Electrochemical Intelligent Recognition of Mineral Materials Based on Superpixel Image Segmentation" was retracted in 2023. Reasons: signs of a paper mill; suspected computer-generated content; unreliable results or conclusions; concerns about the data.

## 5. Conclusion

It is proved that the method of electrochemical intelligent recognition of mineral materials based on superpixel image segmentation is feasible, which effectively solves the problem of time and labor consumption in the manual identification of rock thin sections, meets the needs of geologists for rapid identification of rock thin sections, makes up for the low efficiency of traditional manual identification, and improves the efficiency of identifying rock thin sections. The research and development of automatic identification equipment for rock thin-section samples has high application value. Sandstone is the most common and valuable type of rock slice identification, so the recognition of sandstone slice image is studied. Firstly, the image segmentation technology suitable for sandstone slice image is studied. It is expected to extract the important components in the image through image segmentation, and then the convolution neural network model is designed to identify the material category of each component. In the research process of sandstone slice image segmentation and recognition, three image data sets were collected and produced, and tens of thousands of images were labeled and processed. The data set includes sandstone image segmentation data set used to verify the performance of image segmentation algorithm, rock slice image data set used to train image recognition model, and sandstone particle image recognition data set. According to all the experimental results, after the design of superpixel algorithm and regional merger algorithm, the final sandstone chip image segmentation results are close to the manual annotation results, which is conducive to the subsequent sandstone component identification research. The feasibility of this method is verified.

## Figures and Tables

**Figure 1:** Framework of particle segmentation method for sandstone image.

**Figure 2:** Arbitrary PDF.

**Figure 3:** Uniform PDF.

**Figure 4:** Residual learning module.

**Figure 5:** Comparison of the number of superpixels generated by the algorithm.

**Table 1:** Average time of algorithm.

algorithm	QS	TP	SEEDS	LSC	SLIC	AS-SLIC
Average time	258.93	11.31	0.88	7.09	3.21	7.25

The article "Electrochemical Intelligent Recognition of Mineral Materials Based on Superpixel Image Segmentation" was retracted in 2023. Reasons: signs of a paper mill; suspected computer-generated content; unreliable results or conclusions; concerns about the data.

## Data Availability

The data used to support the findings of this study are available from the corresponding author upon request.
